# Analysis of Effect on Infection Factors and Nursing Care of Postoperative Incision in Gynecological Cancer Patients

**DOI:** 10.1155/2021/2996216

**Published:** 2021-12-06

**Authors:** Yan Sun

**Affiliations:** Department of Gynecology, The First People's Hospital of Lianyungang City, Jiangsu Province, China

## Abstract

**Purpose:**

To study the effect on infection factors and nursing care of postoperative incision in gynecological cancer patients.

**Method:**

72 patients with gynecological malignant tumors who came to the hospital from January 2019 to December 2019 were selected as the research objects. They were divided into the study group and control group by cluster random sampling. The control group was given routine nursing mode, including matters needing attention in surgery, health education, prevention of complications, and dietary guidance. The study group implemented the high-quality nursing mode on the basis of the control group. Postoperative situation, incision infection rate, and quality of life were observed and compared between the two groups.

**Results:**

The control group's time to get out of bed, postoperative eating time, postoperative exhaust time, and hospital stay were longer than those of the study group. The comparison of the postoperative related conditions of the two groups showed that *P* < 0.05, which indicated that the difference was statistically significant. The postoperative incision infection rate in the study group was 2.78%, and in the control group, the postoperative incision infection rate was 19.44%; the postoperative incision infection rate in the study group was significantly lower than that in the control group. The difference was statistically significant, *P* < 0.05. The factors affecting the quality of life of patients in the study group were lower than that of the control group, and the difference was statistically significant, *P* < 0.05. Time to get out of bed, postoperative eating time, postoperative exhaust time, hospital stay, and quality of life were the main influencing factors of postoperative incision infection in gynecological tumors.

**Conclusion:**

Time to get out of bed, postoperative eating time, postoperative exhaust time, hospital stay, and quality of life were the main influencing factors of postoperative incision infection in gynecological tumors. High-quality nursing intervention had better clinical nursing effect in preventing postoperative incision infection. It should be widely used in clinical nursing.

## 1. Introduction

Among gynecological malignant tumors, ovarian malignant tumors and cervical and uterine malignant tumors are the most common [1]. The main clinical treatment for gynecological malignant tumors is surgical resection plus chemoradiotherapy. However, the surgical excision is wide, and the incision is large, Therefore, once postoperative incision infection occurs in gynecological tumor patients, it will not only affect the treatment effect but also increase the burden of treatment. In addition, after radiotherapy and chemotherapy, the body is damaged, the immunity is reduced, and complications are prone to occur in the perioperative period. Incision infection is a common postoperative complication [2, 3]; in severe cases, it can even directly lead to failure of the operation [4, 5]. The influencing factors of postoperative incision infection in gynecological tumor patients were analyzed, and then targeted high-quality nursing intervention programs were developed. It is helpful to improve the curative effect of gynecological tumor surgery [6]. At the same time, nursing intervention is an important way to prevent perioperative infection [7]. Giving targeted nursing intervention before, during, and after surgery can effectively prevent and reduce surgical infection. In this study, 72 patients with gynecological tumors treated by surgery in our hospital from January 2019 to December 2019 were analyzed. This study analyzed the influencing factors of infection and the effect of clinical intervention. The results are summarized and reported as follows.

## 2. Experimental

### 2.1. Normal Information

72 patients with gynecological malignant tumors who came to the hospital from January 2019 to December 2019 were selected as the research objects. They were divided into study group and control group by cluster random sampling. In the study group, 36 patients were aged 31-69 years, with an average age of (46.43 ± 2.29) years. Among them, there were 10 cases of cervical cancer, 14 cases of uterine fibroids, 8 cases of ovarian tumors, and 4 cases of endometrial cancer. 16 patients underwent laparoscopic surgery and 20 underwent open surgery. In the control group, 36 patients were aged 31-70 years, with an average age of (44.28 ± 1.06) years. Among them, there were 10 cases of cervical cancer, 9 cases of uterine fibroids, 11 cases of ovarian tumors, and 6 cases of endometrial cancer. 19 patients underwent laparoscopic surgery and 17 underwent open surgery. The normal information of the two groups of patients were statistically processed. The results showed that *P* > 0.05, with no statistical difference, and this was comparable. Comparison of the normal information was shown in Table 1:

Inclusion criteria: ① age range was 31~70 years old, ② all patients were confirmed by histopathological examination before operation, ③ all underwent surgical treatment, ④ no urinary tract infection was found before the operation, and ⑤ this study was approved by the ethics Committee of the first people's Hospital of Lianyungang City (Approved No. of ethic committee: KQEC-2019-335/32), and the informed consent of the family members and patients was obtained.

Exclusion criteria: ① pregnant and lactating women; ② having an infectious disease; ③ heart, liver, and kidney dysfunction; and ④ received hormone medication before surgery.

### 2.2. Methods

#### 2.2.1. Nursing Measures to the Control Group

The control group was given routine nursing mode, including matters needing attention in operation, health education, prevention of complications, and dietary guidance.

#### 2.2.2. Nursing Measures to the Study Group

For the study group, implementing the high-quality care model on the basis of the control group is as follows: ① formulating rules and regulations, quality care required the guarantee of mandatory rules and regulations, relevant content included work flow and job responsibility, and carrying out assessment regularly to show supervision. ② Updating the nursing model, improving the nursing model on the basis of the original, setting up a nursing team, which included 1 responsible nurse,1 team member, and clarifying the division of nursing care. For patients with severe illness, complex nursing content, and communication difficulties, the responsible nursing with rich nursing experience would be undertaken. For the relatively simple ones, team members were responsible for each patient, and a nurse was responsible for each patient from the beginning to the end. ③ Attention should be paid to preoperative nursing. Reasonable assessment should be made on the nutritional status, blood sugar status, anemia, and complications of patients before surgery. Special care should be given to special patients. For example, for patients with malnutrition or diseases such as hyperglycemia and anemia, not only should they be corrected in a timely manner before surgery but also should focus on strengthening the control after surgery. The incision healing of patients should be regularly observed, and the dressing should be changed on time. ④ Implementing personalized psychological care, carrying out perioperative psychological care and explain related knowledge, the focus of work should be placed on the patient, care details, and nursing staff, and patients should communicate fully, respecting the patient's personal habits, trying to meet the patient's reasonable requirements, and reflecting personalized care. ⑤ Other care measures are as follows: observing closely the patient's vital signs and wound bleeding after surgery, focusing on strengthening the care of patients undergoing open surgery, giving them the necessary nutritional support and encouraging them to carry out early activities, and focusing on strengthening preoperative nursing care for patients with fever; for instance, postponing the operation time, finding out the cause of fever, giving antibiotics to the treatment, and ensuring that the ward was clean and airy.

### 2.3. Observation Indicator

Observing three indicators: ① postoperative conditions, which were including hospital stay, postoperative exhaust time, postoperative eating time, and bedtime activities. ② Incision infection rate is as follows: according to “Diagnostic Criteria for Hospital Infection (Trial)” [8], diagnosing the postoperative wound infection of the patient; the presence of redness, swelling, pain, heat, and purulent discharged from the incision; and patients who had a positive bacterial cultured medium for purulent secretions. All were judged to be incision infection, infection number/case number × 100%. ③ Quality of life: using Nottingham Health Profile (NHP) [9] for assessment, which were including emotion, sleep, pain, energy, physical activity, and social activity, the score was inversely proportional to the quality of life.

### 2.4. Statistical Treatment

The measurement and statistical data in this study were calculated and processed using SPSS19.0. Data verification was performed using (*χ*^2^), using (%) to represent its statistical data. *P* < 0.05 indicated that the difference was statistically significant.

## 3. Results

### 3.1. Postoperative Related Conditions

The control group's time to get out of bed, postoperative eating time, postoperative exhaust time, and hospital stay was longer than those of the study group. The comparison of the postoperative related conditions of the two groups showed that *P* < 0.05, which indicated that the difference was statistically significant. Comparison of postoperative related conditions was shown in Table 2:

### 3.2. Postoperative Incision Infection Rate

The postoperative incision infection rate in the study group was 2.78%, and in the control group, the postoperative incision infection rate was 19.44%; the postoperative incision infection rate in the study group was significantly lower than that in the control group. The difference was statistically significant, *P* < 0.05. Comparison of postoperative incision infection rate was shown in Table 3:

### 3.3. Quality of Life

The factors affecting the quality of life of patients in the study group were lower than that of the control group, and the difference was statistically significant, *P* < 0.05. Comparison of quality of life was shown in Table 4:

### 3.4. Multivariate Logistic Regression Analysis of Postoperative Incision and Nursing Related Infection

Time to get out of bed, postoperative eating time, postoperative exhaust time, hospital stay, and quality of life were the main influencing factors of postoperative incision infection in gynecological tumors. Multivariate logistic regression analysis of postoperative incision and nursing related infection was shown in Table 5:

## 4. Discussion

The detection rate of gynecological malignant tumor is increasing, which is a serious threat to women's life and mental health [10, 11]. Once gynecological tumor is diagnosed, it is difficult for patients to accept it within a short period of time, and they bear great psychological pressure. After the patient begins to accept slowly, the patient worries about the treatment cost of the disease [12], the prognosis after the operation, the adverse reactions brought by chemotherapy, and so on. The common treatment method for gynecological tumors is surgical resection, but this type of surgery, especially for patients with malignant tumors, not only takes longer [13, 14, 15]. And the operation is more complicated, involving many organs, and usually causing great trauma to the patient. In addition, surgical treatment has trauma and incision, and incision infection is a common complication after surgery [16, 17]. Once the incision has symptoms such as redness, swelling, dehiscence, and discharge, it will reduce the treatment effect, affect the prognosis, and prolong the hospital stay. In severe cases, it can cause systemic infection, organ failure, and life threatening. Therefore, to analyze the influencing factors of incisional infection after gynecological tumor operation is of great importance to prevent infection. The prevention of postoperative incision infection is not only related to clinical operation and medication but also plays an important role in nursing intervention [18]. Through this study, it was found that time to get out of bed, postoperative eating time, postoperative exhaust time, hospital stay, and quality of life were the main influencing factors of postoperative incision infection in gynecological tumors. The goal of nursing is “patient satisfaction, social satisfaction, government satisfaction.” The whole nursing process requires nursing staff to provide continuous, satisfactory, and whole-process nursing services. Changing the situation where patients or their families hire nursing workers to make up for the lack of nursing work and improve the nurse-patient relationship [19, 20]. The control group's time to get out of bed, postoperative eating time, postoperative exhaust time, and hospital stay were longer than those of the study group. The comparison of the postoperative related conditions of the two groups showed that *P* < 0.05, which indicated that the difference was statistically significant. The postoperative incision infection rate in the study group was 2.78%, and in the control group, the postoperative incision infection rate was 19.44%; the postoperative incision infection rate in the study group was significantly lower than that in the control group. The difference was statistically significant, *P* < 0.05. The factors affecting the quality of life of patients in the study group were lower than that of the control group, and the difference was statistically significant, *P* < 0.05. Time to get out of bed, postoperative eating time, postoperative exhaust time, hospital stay, and quality of life were the main influencing factors of postoperative incision infection in gynecological tumors. Thus, the measures implemented in the study group were conducive to postoperative recovery and improvement of quality of life. It fully embodied the clinical advantages of high-quality nursing and was in line with the general trend of today's medical reform.

In summary, time to get out of bed, postoperative eating time, postoperative exhaust time, hospital stay, and quality of life were the main influencing factors of postoperative incision infection in gynecological tumors. High-quality nursing intervention in the prevention of postoperative incision infection has a better clinical nursing effect, and it should be widely used in clinical nursing.

## Figures and Tables

**Table 1:** Comparison of the normal information.

Groups	Age		Types of gynecological tumors				Types of surgery	
	Age range	Average age	Cervical cancer	Uterine fibroids	Ovarian tumors	Endometrial cancer	Laparoscopic surgery	Open surgery
Study group	31-69	46.43 ± 2.29	10	14	8	4	16	20
Control group	31-70	44.28 ± 1.06	10	9	11	6	19	17

**Table 2:** Comparison of postoperative related conditions.

Groups	*n*	Time to get out of bed (h)	Time to postoperative eating (h)	Time to postoperative exhaust (h)	Time to hospital stay (h)
Study group	36	38.20 ± 13.72	50.14 ± 8.41	29.27 ± 7.32	8.32 ± 3.64
Control group	36	49.75 ± 12.55	59.28 ± 9.56	36.89 ± 9.61	12.37 ± 4.83
*t*		3.856	4.285	4.106	3.773
*P*		<0.05	<0.05	<0.05	<0.05

**Table 3:** Comparison of postoperative incision infection rate.

Groups	*n*	Number of infections	Infection rate (%)
Study group	36	1	2.78
Control group	36	7	19.44
*χ* ^2^		4.253	5.351
*P*		0.012	0.022

**Table 4:** Comparison of quality of life.

Groups	Study group	Control group	*t*	*P*
Social activity	22.53 ± 2.09	27.75 ± 2.31	4.514	<0.05
Sleep	17.62 ± 1.81	21.29 ± 2.23	4.128	<0.05
Emotion	14.23 ± 1.39	20.14 ± 1.78	4.809	<0.05
Energy	20.70 ± 2.39	26.34 ± 2.77	4.751	<0.05
Pain	24.38 ± 2.59	32.75 ± 2.66	5.613	<0.05
Physical activity	20.32 ± 1.38	28.21 ± 1.75	5.125	<0.05

**Table 5:** Multivariate logistic regression analysis of postoperative incision and nursing related infection.

Influencing factors	*P*	Odds ratio	*β*	95% confidence interval	Wald *χ*^2^
Time to get out of bed	0.003	5.884	1.326	0.879~1.248	17.328
Time to postoperative eating	0.004	5.706	1.508	0.756~1.054	16.088
Time to postoperative exhaust	0.002	6.576	1.604	0.824~1.281	17.822
Time to hospital stay	0.005	15.629	2.317	0.762~1.058	14.301
Quality of life	0.000	17.870	2.415	0.729~1.162	22.021

## Data Availability

The datasets used during the present study are available from the corresponding author upon reasonable request.

## References

[1] Barcellini A., Vitolo V., Facoetti A. (2019). Feasibility of carbon ion radiotherapy in the treatment of gynecological Melanoma. *In vivo*.

[2] Akazawa M., Onjo S. (2018). Malignant transformation of mature cystic teratoma: is squamous cell carcinoma different from the other types of Neoplasm?. *International Journal of Gynecological Cancer*.

[3] Wolsky R., Price M. A., Zaloudek C. J., Rabban J. T. (2018). Mucosal proliferations in completely examined fallopian tubes accompanying ovarian low-grade serous Tumors. *International journal of gynecological pathology: Official journal of the International Society of Gynecological Pathologists*.

[4] Hanayneh W., Starr J., George T., Parekh H. (2018). Extragastrointestinal stromal tumors of the pelvic cavity and the vagina: Two case reports and review of the literature. *Oncology Reports*.

[5] di Donato V., Iacobelli V., Schiavi M. C. (2018). Impact of hormone receptor status and Ki-67 expression on disease-free survival in patients affected by high-risk endometrial cancer. *International Journal of Gynecological Cancer*.

[6] Mohr-Sasson A., Machtinger R., Mashiach R. (2019). Long-term outcome of MR-guided focused ultrasound treatment and laparoscopic myomectomy for symptomatic uterine fibroid tumors. *Obstetrical & Gynecological Survey*.

[7] Kalantari S. (2020). Nursing care from the human caring theory lens in a female breast cancer patient: a care case study. *entific Journal of Nursing Midwifery and Paramedical Faculty*.

[8] Headquarters (2003). Diagnostic criteria for hospital infection (Trial). *Modern Practical Medicine*.

[9] Teixeirasalmela L. F. (2014). *Nottingham Health Profile (NHP)[M]*.

[10] Torre-Montero J. C. D. L. (2019). Gynecological cancer. *Principle of Nursing in Oncology*.

[11] Naef R., Kaeppeli B. M., Lanter R., Petry H. (2020). Implementing family systems care through an educational intervention with nurses and midwives in obstetrics and gynecological care: a mixed-methods evaluation. *Journal of family nursing*.

[12] Gut A., Moch H., Choschzick M. (2018). SOX2 Gene amplification and overexpression is linked to HPV-positive vulvar carcinomas. *International Journal of Gynecological Pathology*.

[13] Alessi A., Pappalardi B., Cerrotta A., Calareso G., Crippa F. (2020). T-staging and target volume definition by imaging in GYN tumors. *Imaging and Interventional Radiology for Radiation Oncology*.

[14] Taurin S., Yang C., Reyes M. (2018). Endometrial cancers harboring mutated fibroblast growth factor Receptor 2 protein are successfully treated with a new small tyrosine kinase inhibitor in an orthotopic mouse Model. *International Journal of Gynecological Cancer*.

[15] Venturella G., Saporita P., Gargano M. L. (2019). The potential role of medicinal mushrooms in the prevention and treatment of Gynecological Cancers: A Review. *International Journal of Medicinal Mushrooms*.

[16] Colpaert R. M., Ramseyer A. M., Luu T., Quick C. M., Frye L. T., Magann E. F. (2019). Diagnosis and management of placental mesenchymal disease. A review of the Literature. *Obstetrical & Gynecological Survey*.

[17] Asano H., Fukano H., Shinozuka N. (2020). Postoperative shock as independent factor for incisional surgical site infection in left-side colorectal perforation. *SN Comprehensive Clinical Medicine*.

[18] Wilson B. R., Sterrett M., Metzinger D., Greer K. E., Gunaratnam B., Medlin E. E. (2019). Postoperative incisional cryoanalgesia for robotic hysterectomy. *Gynecologic Oncology*.

[19] Cruickshank S. (2019). The changing reality of cancer nursing care. *Cancer Nursing Practice*.

[20] Hudson J., Reblin M., Clayton M. F., Ellington L. (2019). Addressing cancer patient and caregiver role transitions during home hospice nursing care. *Palliative & Supportive Care*.

